The article "IoT-Based Hybrid Ensemble Machine Learning Model for Efficient Diabetes Mellitus Prediction" was retracted in 2023. Reasons: unreliable results or conclusions; lack of ethics approval or compliance; concerns about the data; concerns about the peer review.

# IoT-Based Hybrid Ensemble Machine Learning Model for Efficient Diabetes Mellitus Prediction

**DOI:** 10.1155/2022/2389636

**Published:** 2022-05-18

**Authors:** Sasmita Padhy, Sachikanta Dash, Sidheswar Routray, Sultan Ahmad, Jabeen Nazeer, Afroj Alam

**Affiliations:** ^1^School of Computing Science and Engineering, VIT Bhopal University, Bhopal, Madhya Pradesh, India; ^2^Department of Computer Science and Engineering, GIET University, Gunupur, Odisha, India; ^3^Department of Computer Science and Engineering, School of Engineering, Indrashil University, Rajpur, Mehsana, Gujarat, India; ^4^Department of Computer Science, College of Computer Engineering and Sciences, Prince Sattam Bin Abdulaziz University, Alkharj 11942, Saudi Arabia; ^5^Department of Computer Science, Bakhtar University, Kabul, Afghanistan

## Abstract

Nowadays, there is a growing need for Internet of Things (IoT)-based mobile healthcare applications that help to predict diseases. In recent years, several people have been diagnosed with diabetes, and according to World Health Organization (WHO), diabetes affects 346 million individuals worldwide. Therefore, we propose a noninvasive self-care system based on the IoT and machine learning (ML) that analyses blood sugar and other key indicators to predict diabetes early. The main purpose of this work is to develop enhanced diabetes management applications which help in patient monitoring and technology-assisted decision-making. The proposed hybrid ensemble ML model predicts diabetes mellitus by combining both bagging and boosting methods. An online IoT-based application and offline questionnaire with 15 questions about health, family history, and lifestyle were used to recruit a total of 10221 people for the study. For both datasets, the experimental findings suggest that our proposed model outperforms state-of-the-art techniques.

## 1. Introduction

Diabetes, often known to be diabetes mellitus (DM), is a group of metabolic illnesses characterized by persistently elevated blood sugar levels. Excessive urination, continuous thirst, and an increase in hunger are all symptoms of high blood sugar [1]. Diabetes, if not treated promptly, can lead to significant health problems in a person, such as hyperglycaemic, hyperosmolar condition, diabetic ketoacidosis, or even one of the results for death. Long-term effects include stroke, cardiovascular disease, foot ulcers, renal failure, and vision problems [2]. When the body's pancreas is unable to produce enough insulin, diabetes develops, or even if the insulin generated is not appropriately used by the body's cells and tissues. The diabetes mellitus can be categorized into the following three types [3].

- “Insulin-subordinate diabetes mellitus” (ISDM) is a disorder in which the pancreas produces less insulin than the body demands, resulting in type 1 diabetes. To compensate for the pancreas' lower insulin production, type 1 diabetics require supplementary insulin.
- Type-2 diabetes is defined as an insulin resistive body, which occurs when the body's cells react to the insulin differently than they would ordinarily. “Adult starting diabetes” or “noninsulin subordinate diabetes mellitus” (NISDM) is other term for this condition. This kind of diabetes is more common in those with a high BMI or who have a sedentary lifestyle.
- During the time of pregnancy, the third type of diabetes called gestational diabetes may develop.

A typical human's sugar levels may vary from range 70 to 99 mg/dL. A person is classified as having diabetes when her or his fasting glucose level reached 126 mg/dL. From the healthcare point of view, someone with a higher glucose level between 100 and 125 mg/dL may be considered prediabetic [4]. In such an individual, type 2 diabetes is more prone to develop. GDM (gestational diabetes mellitus) is a kind of diabetes that develops during pregnancy that is no clear evidence of diabetes during the 2nd and 3rd trimesters of pregnancy. Diabetic may be caused by other factors, such as monogenic diabetes syndromes, and exocrine pancreas diseases.

Diabetes disorders have the capacity to harm several sections of the human body. The followings are some of the human body components that are impacted by diabetes: the heart, the eye, the kidney, and the nerves of humans [5, 6]. As the name implies, it is simple to estimate how much chronic and serious illnesses shorten human life. Machine learning algorithms have varying degrees of categorization and prediction capacity [7]. According to [8], no one strategy is superior in terms of performance and accuracy for all diseases; although one classifier performs best in a certain dataset, another method or approach outperforms the others for other diseases. The new or proposed study focuses on a novel combination or hybridization of multiple classifiers for diabetic mellitus (DD) classification and prediction, solving the difficulty of single or individual classifiers. The new study proposes using several machine learning methods (MLTs) to detect diabetic mellitus (DM) at an early stage in order to save human lives. The major goal of this research is to create an information system that can forecast diabetes with greater accuracy.

### 1.1. Symptoms

The symptoms of diabetes may vary depending on the blood glucose level. Some people, particularly those with type-2 diabetes or prediabetes, may not show any signs at all. Symptoms of type-1 diabetes appear more quickly and are more severe. Some of the signs and symptoms of type 1 and type 2 diabetes are as follows:

- Availability of ketones in urine
- Thirst rises
- Frequent urination
- Hunger to the point of death
- Frequent weight loss
- Fatigue
- Cloudy vision
- Long-lasting sores
- Infections that recur often, such as gum or skin infections, as well as vaginal infections
- Obesity is defined as a BMI greater than 25

Diabetes is a familial disease that affects several members of the family. People have HDL cholesterol levels of less than 40 milligrams per deciliter in their blood. People with polycystic ovary syndrome over 45 years old from ethnic groupings such as African Americans, Native Americans, Latin Americans, and Asian Pacific live a sedentary lifestyle.

The IoT in genetic terms is used for a collection of connected bodily objects that may be accessed over the Internet. The “thing” in the Internet of Things can be an object with sensors that have been assigned an IP address [9]. It can build and share data over a network without requiring any human assistance. Individuals are becoming increasingly conscious of and committed to their own health. A large portion of hospital expenditures is spent on medical examinations. There is an unrivaled opportunity to improve the quality of care and the efficacy of therapies by adopting technology-based healthcare procedures [10–13].

There are a variety of advantages to implementing IoT, including real-time applications and data collection and analysis.  Figure 1 depicts how this significant shift in medical practice will be examined in an IoT hospital. An ID card will be issued to a diabetic patient that, once scanned, will help to connect them to a secure cloud where their electronic health-related data and medical records would be stored. On a tablet or computer, doctors and attendants will have no trouble using the record.

The remainder of the paper is laid out as follows: Section 2 focuses on the related work reviewed during the proposed work.  Section 3 briefly describes the traditional models which were implemented for prediction and comparison. In section 4, the proposed methodologies along with the implementation are presented, and experimental results along with a discussion are carried out in section 4. Lastly, the conclusion of the proposed work is presented in section 5.

## 2. Related Work

Diabetes may be a major disease, with an affected adult population of more than 70%. To anticipate diabetes symptoms, several researchers have utilized approaches such as data mining and machine learning [14]. Only a handful has utilized both neural networks and genetic algorithms. Because diabetes prediction is a supervised problem, supervised techniques such as machine learning, data mining, and artificial neural networks have been employed by numerous researchers.

Numerous scientific researchers have utilized the Pima Indians dataset for diabetes (PIDD) to predict diabetes. Weka and machine learning approaches were used in [15–17]. Data mining, machine learning, neural network, and hybrid techniques are among the methodologies used by researchers. In diabetes prediction, artificial neural networks (ANN) are commonly employed. Komi et al. [18] described several data mining approaches that were used for showing information for type 2 diabetes. Swapna et al. [19] used electrocardiogram (ECG) data to detect diabetes using deep learning algorithms. They retrieved features using a convolution neural network (CNN), and then, a support vector machine algorithm is used to extract the features. Finally, they determined that the accuracy rate was 95.7%. To represent knowledge-based systems, fuzzy cognitive maps (FCM) have been used. Tuppad et al. [20] proposed a strategy for predicting gestational diabetes using the case-based fuzzy cognitive maps decision-making system. Saeedi et al. [8] proposed a framework to detect the presence or absence of diabetes mellitus. This framework is based on a delicate registering technique, specifically fuzzy cognitive maps (FCM). The product instrument was tested on 50 cases, with 96% accuracy in predicting outcomes.

A significant advancement in medical imaging technology has occurred in the last decade as a result of the application of iris image detection. Furthermore, the machine learning approaches are useful to improve the determining capacity of iridologists. Systemic disease with ocular consequences was linked to the proposed model [21]. The random forest classifier achieved 89.66% accuracy by analyzing 200 subject data from 100 diabetic and nondiabetic people. To predict diabetes using PIDD, Sisodia et al. [22] utilized three machine learning algorithms: decision tree (DT), support vector machine (SVM), and naive Bayes (NB). The accuracy of 76.3 percent was determined for the naive Bayes classifier. Wu et al. [23] employed a data mining technique to determine an individual's development of risk factors for type-2 diabetes with an accuracy of 95.42%. Experimentally, the initial seed point value resulted in the modification. Choubey et al. [24] utilized J48, random forest, and ANN for classification and utilising unsupervised techniques like principal component analysis (PCA) after feature reduction.

Siddiqui et al. wanted to see if there was a link between diabetes and metabolic syndrome [25]. For forecasting, the authors employed the Naive Bayes and J48 decision tree models. The training set was balanced by using k-medoids sampling. In their study, NB surpassed the competition. The effects of different machine learning techniques on the determination of diabetes are summarized by Wittenbecher et al. [26] and Zhou et al. [27]. The proposed work first records the patient information through sensors and then transmitted it to the cloud server. The proposed concept got a 0.045 correlation coefficient value which increases the strength of the algorithm [28].

All age groups finally saw a linear connection between BMI and diabetes. BMI and age were shown to be good predictors of diabetes risk. Zou et al. [29] developed a nomogram based on the seven diabetes risk factors to help people predict their type 2 diabetes risk. A robot is intelligent in the sense that it has built-in watching and detecting capabilities, as well as the ability to gather sensor data from various sources and fuse it for the device's “acting” purpose. Mall et al. [30] introduced the e-health mind stage by employing robots that were connected via IoT to provide personalized varied care methods, particularly to diabetes patients. The robot is equipped with sensors that monitor the diabetic's medical and dietary status, providing them with comprehensive multidimensional care.

According to statistical analysis and the multivariate Cox regression method [31], the TG/HDL-C ratio was positively associated with the prevalence of diabetes in the Chinese population. The author proposed an MSSO-ANFIS model for the diagnosis of heart disease which uses a levy flight algorithm. The proposed model obtains 99.45 accuracies and 96.54 precision [32]. It is concluded that those in their 30s and 40s with elevated ALT (alanine aminotransferase) are at a higher risk than those with low ALT. Choi et al. [33] employed machine learning (ML) algorithms on people with nondiabetics and a high risk of cardiovascular disease. In this paper, the author proposed an MDCNN classifier that collects data from IoT sensors. The proposed model obtains 98.2 accuracies as compared with existing classifiers [34]. Over the last five years, Korea University Guro Hospital has accumulated data in the form of an EMR (electronic medical record) [35]. Various ML methods were then employed with the help of cross-validation. The most accurate model is the logistic regression model [36–38].

## 3. Different Machine Learning Approaches

Once the data are available, we use machine learning techniques to analyze it. We use a number of classification algorithms to predict diabetes. The strategies were tested using a diabetic dataset from Pima Indians. The major purpose is to assess the results of these methods and determine their validity, as well as who was accountable, using machine learning techniques. This is a crucial characteristic that plays a big part in prediction. The methods are as follows.

### 3.1. Logistic Regression (LR)

The sigmoid function is used to evaluate probabilities in LR, which is a sort of supervised learning method. The sigmoid function calculates the relationship between at least one independent variable and a binary-dependent variable. The LR model is a form of machine learning classification model that has binary values like 0 or 1, −1 or 1, true or false as the dependent variable and the independent variable such as interval, ordinal, binominal, or ratio level. The logistic/sigmoid equation function is as follows:

(1) $$\begin{array}{c} y=\frac{1}{1+e^{-x}}, \end{array}$$

where *y* is denoted as the outcome of the weighted sum with variables *x* as input. Here, the output is estimated as 1 if it is more than 0.5; else, it is 0.

### 3.2. Support Vector Machine

Out of many supervised classification techniques, the SVM is one of them that may be used for regression and classification in machine learning techniques. It is mostly used to solve classification difficulties. The main goal of SVM is to categorize the data point using a suitable hyperplane in a multidimensional space. A hyperplane is considered as a boundary of classification for data values. In this technique, each data item in n-dimensional space is represented as a point, with the value of each feature matching the value of a certain coordinate. We would plot these two components in two-dimensional space, with two layouts for each point if we only knew two qualities about an individual, such as height and hair length (these directions are known as support vectors). Because the two closest focuses are the furthest distance from the line in Figure 1, the dark line divides the data into two different organized groupings. Our classifier is represented by this line. Based on the falling of testing data on both sides of the line, the new data are able to be categorized into one of two categories.

### 3.3. K-Nearest Neighbor

Both regression and classification issues may be solved using the K-nearest neighbor (KNN) technique [39]. However, in the industry, it is more commonly utilized in classification issues. KNN is a straightforward computation that stores all existing examples and ranks new ones based on the votes of its *k* neighbors. To place the case in the class with the most people among its K nearest neighbors, distance work is used. The Manhattan, Hamming, Euclidean, and Makowski distances are among the distance capabilities. The first 3 numbers of features are used for indefinite functions, whereas the 4th one is used for absolute variables. If *K* = 1, the case is essentially assigned to the class of the next closest neighbor. Selecting K for KNN modeling might be challenging at times.

### 3.4. Random Forest

The random forest (RF) classifier technique generates several decision trees from a portion of the randomly chosen dataset used for training purposes. The votes from several decision trees are combined to establish the final class of test items [29]. Each tree offers a classification to a new object based on characteristics, and for that class, we say the tree as “votes.” The classification employing the utmost votes is selected by the forest. The random forest has several options that produce accurate predictions for a variety of applications. The following is how each tree is planted and grown:

1. If N instances are there in the training set then, an *N* cases random sample is chosen with replacement and that can be utilized for training the tree.
2. If there are *M* inputs and out of which *m* inputs are randomly chosen at each node out of the *M* variables, where *m* < *M*, with the finest split on this input *m* being utilized to divide the node. Here, *m* is kept constant throughout the growth of the forest.
3. Every tree is brought to its full potential. Pruning is out of the question.

## 4. Proposed Methodology

A total of 10221 individuals aged 18 and above were chosen for this study, including 6031 men and 4190 females. The participants were invited to complete an online IoT sensing operation and a questionnaire (Table 1) that they had developed themselves based on the factors that might contribute to diabetes. The same tests were carried out on another database, the PIMA Indian Diabetes database [31–33], to validate the model's validity.  Figure 2 depicts a sample dataset gathered by a questionnaire.

### 4.1. M-Health Systems Using Web-Based IoT Service and Sensors for Diabetes Monitoring

When the reading rises, an update automatically is sent to the doctor via voice calls or text messages. This may be accomplished through the use of a web application that establishes worldwide communication between the patient's online portal and the IoT sensor of the patient, which updates the patient's personal information such as blood sugar level and remaining medicines. This is one method for managing diabetes remotely that has been proposed.

One of the most extensively utilized technologies is using IoT devices to monitor diabetes patients. By just registering in the programme that talks with the IoT sensors, one may keep track of their diabetes state. This application simplifies the monitoring process for new members, diabetes patients, their family members, and anybody else who is interested. The user must have their user name and password. After the member's information has been verified and the registration has been completed, the user may log in and access the extra services that are offered. It is vital to keep track of the user profile that was generated when you signed up. It is vital that their sensor readings be automatically enrolled. Here, the RFID tag must be linked with the sensors that are attached to the patient. The IoT can keep track on the patient remotely irrespective of the availability of the patient either in the home or at the hospital. A number of sensors are used in this technique. Arduino is an open-source microcontroller that makes things more flexible and accessible, allowing you to develop transdisciplinary projects. Body temperature sensors, OPS2 (oxygen and pulse sensor), and blood pressure sensors are all examples of e-health sensors that use Arduino. A glucometer sensor is a medical gadget that measures glucose levels in the blood. By pricking the skin with a lancet, a small drop of blood is sufficient to compute the level of blood sugar in the patient.

All the above-mentioned sensors must be linked to the body of the patient so that the necessary detailed reading of the patient can be monitored by the e-health sensor. The login credentials of the patient are verified whenever the patient logged in using an RFID tag. The patients' detailed data are then immediately updated. Sensors affixed to the body take the readings, which are then connected utilising IoT tools. It will immediately send a message or a phone call to the patient's doctor regarding the details condition of the patient. The data are subsequently entered into a diabetic patient management website. In Figure 3, the different sensors used to monitor the patient and record their information for further prediction are depicted.

Once the data are collected through the IoT sensor and questionnaires, we applied a hybrid bagging and boosting, ensemble methodology to the data. The proposed work is divided into two stages. During the first stage, the training data are fit into three different traditional machine learning models which are logistic regression, K-nearest neighbor, and support vector machine individually. Then, a voting process is applied to the resultant prediction which elects the output among them. This whole process is known as bagging. In the second stage, the identified output is then fit through the random forest model to boost the prediction. This process is known as boosting. The detailed flow of the proposed model is presented in Figure 4.

### 4.2. Implementation

The study's implementation was done with Google Colab, and the coding was done with the python programming language. Both the Pima dataset and the gathered dataset were used to forecast the availability of diabetes. After then, each classifier's predictions are compared with the proposed model.

### 4.3. Available Pima Dataset

Parameters used in Pima datasets are as follows:

1. Age
2. Glucose
3. Blood pressure
4. BMI
5. Insulin
6. Skin thickness
7. Diabetes pedigree function
8. Pregnancies
9. Outcome

## 5. Experimental Results and Discussions

The data set used to predict diabetes is shown in Tables 2 and 3. The diabetes parameters serve as the variable, which is dependent, whereas the other factors served as independent ones. For dependent diabetes features, only two values are accepted, with a “zero” indicating no diabetes and a “one” signifying the availability of diabetes. The whole sample is divided into two groups, with a ratio of 70 : 30 for the training and testing dataset. All four methods of classification were used for prediction. The training data were then used to predict the test set outcomes using SVM, k-nearest neighbor, RF, and LR classifications, resulting in the confusion matrix given in Table 2.

The measure provided in equations (2)–(8) may be computed using the obtained confusion matrices. True Negative (TN), True Positive (TP), False Negative (FN), and False Positive (FP) were the results of these matrices (TP). Because there are more nondiabetic cases than diabetic cases in both datasets, the TN is greater than the TP. As a consequence, all of the techniques provide positive results. The following measurements have been calculated using the following formulae [34] to determine the precise accuracy of each method:

(2) $$\begin{array}{c} \text{Precision}=\frac{TP}{TP+FP}, \end{array}$$

(3) $$\begin{array}{c} \text{Sensitivity}=\frac{TP}{TP+FN}, \end{array}$$

(4) $$\begin{array}{c} \text{Specificity }=\frac{TN}{TP+FP}, \end{array}$$

(5) $$\begin{array}{c} MCC=\frac{\left(TP*TN\right)-\left(FP+FN\right)}{\sqrt{\left(TP+FP\right)\left(TP+FN\right)\left(TN+FP\right)\left(TN+FN\right)}}, \end{array}$$

(6) $$\begin{array}{c} \text{Error Rate}=\frac{FN\;+FP}{TP+TN+FN+FP}, \end{array}$$

(7) $$\begin{array}{c} F-\text{Measure}=\frac{2*\left(\text{Precision}*\text{Sensitivity}\right)}{\text{Precision }+\text{Sensitivity}}, \end{array}$$

(8) $$\begin{array}{c} \text{Accuracy}=\frac{TN\;+TP}{TP+TN+FN+FP}. \end{array}$$

Another finding is that the accuracy level as per Table 3 among all individual techniques is higher on our collected dataset than on the used PIMA dataset, owing to the former's greater number of variables relevant to assessing diabetes risk. The random forest classifier outperforms all others in terms of accuracy (98.4%), sensitivity, specificity, precision, and F-measure, proving that it is the best technique for our dataset. Furthermore, in the case of random forest, the AUC value is 1, indicating that this model performs exceptionally well in classification.  Figure 5 depicts the clear graph for the ROC curve and AUC for both the collected dataset and PIMA datasets. Here, it indicates that in both cases, the ensemble RF boosting classifier gives the highest result with a value of 1.

The significance of each parameter in the dataset is depicted in Table 4. On the classifier model construction, the python function “summary” is used to perform this analysis. The star beside each parameter indicates the significance of that variable. The ratings are in the following order: where “^∗∗∗^” denotes the highest priority, “^*∗*^” denotes the least important, and a feature without any symbol denotes the least concerned with diabetes.  Figure 6 depicts the correlation matrices of the different parameters, and Figure 7 depicts the comparison of different classification algorithms. There is no statistical significance for the variable with no rating. Variable importance is studied to find which parameter has the greatest impact on the forecast.

### 5.1. Comparative Analysis

Table 5 shows a comparison between the current state of the art and our suggested technique. The author of [19] employed deep learning algorithms to predict diabetes, providing a maximum accuracy of 95.7 percent. Bhatia et al. [6] employed a more accurate genetic algorithm fuzzy cognitive maps and achieved an accuracy of 96 percent. Samant et al. [21] used an improvised random forest technique to achieve 89.66 percent accuracy, whereas Sisodia et al. [22] used modified machine learning algorithms with efficient coding to get 76.3 percent accuracy. Wu et al. [23] have employed improved data mining techniques to get an accuracy of 95.42 percent. Our method achieved a 98.4 percent accuracy by utilising an IoT-based hybrid ensemble machine learning model that is superior to the current state of the art.

## 6. Conclusion

One of the most pressing worldwide health concerns is detecting diabetes risk at an early stage. Our research aims to build up a system for predicting the risk of diabetes mellitus. Three traditional machine learning techniques and the proposed hybrid ensemble model for classification were used in this work, and the results were compared to several statistical metrics. The prediction has been done using ML algorithms on collected 15 diabetes-related data from IoT sensors as well as questionnaires. Also, the four algorithms were used on the PIMA database for prediction. The accuracy level of the proposed classification in our dataset is 98.4 percent, which is the greatest among the others, according to the testing results. For the PIMA dataset, the proposed model also provides the greatest accuracy. All described models generated appreciable results for different parameters such as accuracy and recall sensitivity using four different machine learning methods. It is observed from the results that among all factors, “age,” “family_history,” “physical_activity,” and “regular_intake_of_medicine” have the highest significance. These variables have a larger influence on diabetes prediction than the others. This result can be used to forecast any other illness in the future. This study is currently researching and improving various ML approaches for forecasting diabetes along with other health conditions.

## Figures and Tables

**Figure 1:** Health monitoring in IoT hospitals.

**Figure 2:** Screenshot of the collected dataset.

**Figure 3:** Sensors and services for diabetes monitoring.

**Figure 4:** Flow of the proposed model.

**Figure 5:** (a) ROC curve with AUC for PIMA dataset. (b) ROC curve with AUC for the collected dataset.

**Figure 6:** Correlation matrix.

**Figure 7:** Comparison of traditional classification models and proposed model when implemented on the collected dataset and PIMA dataset.

**Table 1:** Possible answers for different features.

Sl. No	Features	Possible answers
1	Age	More than 18 years
2	Gender	Male 643, Female 429
3	Family history	Yes/No
4	Physical_Activity	1. More_than_one_hour 2. Less_than_one_hour 3. Never
5	Urination_Frequency	1. Frequently 2. Not much
6	Junc_Food_Consumption	Yes/No
7	Blood_Pressure	1. Normal 2. High 3. Low
8	BMI	Numeric
9	Diabetes	Yes/No
10	Reglar_Intake_Of_Medicne	Yes/No
11	No_Of_Pregnancies	Numeric
12	Smoking	Yes/No
13	Alcohol_Consumption	Yes/No
14	Hour_Of_Sleep	Numeric
15	Stress	Yes/No

**Table 2:** Matrix of confusion for different classification methods.

Dataset/Models	Logistic regression	K-nearest neighbor	Support vector machine	Proposed model
PIMA dataset	[[138 12] [42 41]]	[[132 20] [39 44]]	[[143 9] [47 36]]	[[128 20] [36 45]]
Collected dataset	[[192 24] [15 87]]	[[164 38] [46 74]]	[[195 15] [24 93]]	[[224 3] [4 95]]

**Table 3:** Comparison of statistical measurement for various classification techniques.

	Logistic regression		K-nearest neighbor		Support vector machine		Proposed model	
	Collected dataset	Pima dataset	Collected dataset	Pima dataset	Collected dataset	Pima dataset	Collected dataset	Pima dataset
Accuracy	0.872	0.744	0.739	0.708	0.888	0.744	0.984	0.750
Error	0.127	0.255	0.261	0.291	0.112	0.255	0.016	0.250
Sensitivity	0.923	0.775	0.778	0.748	0.898	0.775	0.987	0.789
Specificity	0.764	0.666	0.702	0.603	0.816	0.666	0.916	0.661
Precision	0.885	0.856	0.816	0.832	0.933	0.856	0.991	0.840
F-measure	0.903	0.813	0.797	0.787	0.915	0.813	0.989	0.813
MCC	0.732	0.416	0.503	0.331	0.764	0.416	0.963	0.436
Kappa	0.727	0.470	0.516	0.419	0.713	0.466	0.922	0.488
AUC	0.908	0.765	0.916	0.815	0.893	0.771	0.984	0.978

**Table 4:** Importance of parameters.

	Count	Mean	Std	min	0.25	0.5	0.75	Max
Age^∗∗∗^	10221	32.9026	11.09011	21.00000	24.00000	29.50000	40.00000	66.00000
Gender^∗∗^	10221	0.50649	0.50158	0.00000	0.00000	1.00000	1.00000	1.00000
family_history^∗∗∗^	10221	0.29220	0.45626	0.00000	0.00000	0.00000	1.00000	1.00000
physical_activity^∗∗∗^	10221	1.38311	0.78547	0.00000	1.00000	2.00000	2.00000	2.00000
Regular_intake_of_medicine^∗∗∗^	10221	0.26623	0.44343	0.00000	0.00000	0.00000	1.00000	1.00000
No_of_pregnancies^∗∗^	10221	1.88311	3.08686	0.00000	0.00000	0.00000	3.00000	14.00000
Smoking	10221	0.07792	0.26892	0.00000	0.00000	0.00000	0.00000	1.00000
alcohol_consumption	10221	0.33766	0.47445	0.00000	0.00000	0.00000	1.00000	1.00000
hour_of_sleep^*∗*^	10221	6.59740	0.91836	6.00000	6.00000	6.00000	8.00000	8.00000
Stress	10221	0.44805	0.57214	0.00000	0.00000	0.00000	1.00000	2.00000
Urination_frequency	10221	0.40909	0.49327	0.00000	0.00000	0.00000	1.00000	1.00000
Junc_food_consumption	10221	0.52597	0.50095	0.00000	0.00000	1.00000	1.00000	1.00000
Blood_pressure^∗∗^	10221	0.86363	0.80900	0.00000	0.00000	1.00000	2.00000	2.00000
BMI	10221	32.3701	7.40424	0.00000	28.00000	33.00000	36.00000	67.00000
Diabetes	10221	0.44155	0.49819	0.00000	0.00000	0.00000	1.00000	1.00000

**Table 5:** Comparison study of our suggested work with the current state of the art in terms of accuracy.

Author(Year)	Method	Accuracy (%)
Swapna et al. [19] (2018)	Deep learning algorithms	95.7
Bhatia et al. [6] (2019)	Fuzzy cognitive maps	96
Samant et al. [21] (2017)	Improvised random forest technique	89.66
Sisodia et al. [22] (2018)	Modified machine learning algorithms	76.3
Wu et al. [23] (2018)	Improved data mining techniques	95.42
Our approach	IoT-based hybrid ensemble machine learning model	**98.4**

## Data Availability

The data used to support the findings of this study are available from the author upon request (pinky.sasmita@gmail.com).
